The article "Audience Evaluation and Analysis of Symphony Performance Effects Based on the Genetic Neural Network Algorithm for the Multilayer Perceptron (GA-MLP-NN)" was retracted in 2023. Reasons: suspected computer-generated content; unreliable results or conclusions; concerns about the data; concerns about the results or conclusions.

# Audience Evaluation and Analysis of Symphony Performance Effects Based on the Genetic Neural Network Algorithm for the Multilayer Perceptron (GA-MLP-NN)

**DOI:** 10.1155/2021/4133892

**Published:** 2021-10-08

**Authors:** Cong Yan

**Affiliations:** Shanghai Conservatory of Music, Shanghai 200031, China

## Abstract

Traditional symphony performances need to obtain a large amount of data in terms of effect evaluation to ensure the authenticity and stability of the data. In the process of processing the audience evaluation data, there are problems such as large calculation dimensions and low data relevance. Based on this, this article studies the audience evaluation model of teaching quality based on the multilayer perceptron genetic neural network algorithm for the data processing link in the evaluation of the symphony performance effect. Multilayer perceptrons are combined to collect data on the audience's evaluation information; genetic neural network algorithm is used for comprehensive analysis to realize multivariate analysis and objective evaluation of all vocal data of the symphony performance process and effects according to different characteristics and expressions of the audience evaluation. Changes are analyzed and evaluated accurately. The experimental results show that the performance evaluation model of symphony performance based on the multilayer perceptron genetic neural network algorithm can be quantitatively evaluated in real time and is at least higher in accuracy than the results obtained by the mainstream evaluation method of data postprocessing with optimized iterative algorithms as the core 23.1%, its scope of application is also wider, and it has important practical significance in real-time quantitative evaluation of the effect of symphony performance.

## 1. Introduction

At present, most of the research processes of orchestral performance effect evaluation are based on the traditional “performance type and melodic characteristics research and vocal appreciation” type, supplemented by the “performance audience evaluation” research [1]. In recent years, with the rapid development and popularization of symphonic music, the intelligent analysis mode of symphonic performance effect has become more and more important and has become an important reference index for symphony orchestras [2]. The diversification, comprehensiveness, and quantitative characterization of symphonic performance analysis models have become the mainstream evaluation goals nowadays [3]. At present, the existing orchestral performance effect evaluation is mainly divided into two modes: qualitative evaluation and quantitative evaluation [4]. However, qualitative evaluation has problems such as large errors and subjective factors, while quantitative evaluation can be well controlled in terms of evaluation accuracy, but it has the problem of high evaluation requirements in terms of setting accuracy rules [5]. How to effectively combine quantitative evaluation and qualitative evaluation has become the mainstream direction of research in evaluating the effect of symphony performance [6].

The article "Audience Evaluation and Analysis of Symphony Performance Effects Based on the Genetic Neural Network Algorithm for the Multilayer Perceptron (GA-MLP-NN)" was retracted in 2023. Reasons: suspected computer-generated content; unreliable results or conclusions; concerns about the data; concerns about the results or conclusions.

The innovation of this paper is that the multilayer perceptron genetic neural network algorithm is used in the evaluation of symphony performance. On this basis, it can make full use of a large amount of symphony performance data and extract appropriate symphony performance information from it. Data quantification, information extraction, and analysis of the audience's facial expression changes, emotional performance, and so forth are carried out dynamically to achieve an overall closeness in the audience evaluation data. Compared with the current mainstream performance evaluation methods of data analysis and postprocessing, the symphony performance evaluation management and analysis model proposed by this research uses multitransformed neural network factors to quantitatively describe the quantitative characterization characteristics of different performance processes. The degree of agreement between the similarity of the dimensional vocal analysis model and the expected evaluation index is to complete the ranking of the influence on the performance melody with the quantitative index, which can efficiently analyze the characteristics of the factors that affect the performance of the symphony.

This paper investigates the normalization scheme of audience evaluation and analysis of orchestral performance effects and is divided into five sections.  Section 1 introduces the background of this study and the overall framework.  Section 2 introduces the related work on audience evaluation and analysis of orchestral performance effects.  Section 3 constructs a quality evaluation model of symphony performance analysis mode based on multilayer perceptron genetic neural network algorithm and objective evaluation method and adopts a multilayer perceptron neural network factor method to construct an evaluation index system of symphony performance effect analysis mode.  Section 4 conducts experimental analysis and verification of the quantitative indexes of the orchestral performance effect audience evaluation and analysis model.  Section 5 concludes the work and proposes some findings.

## 2. Related Work

It is known that it is relatively backward in symphony performance analysis model innovation and quality evaluation using computer techniques [7]. At present, some scholars are paying attention to this field. Reed et al. [8] stated that capturing musical performances for virtual reality (VR) is of growing interest to engineers, cultural organizations, and the public, and using VR technique enables perception and localization of sound sources within 3D space. Wu et al. [9] designed the open symphony to explore audience-performer interaction in live music performances, assisted by digital technology, and audiences can conduct improvised performances by voting for various musical modes. Schedl et al. [10] first identified what they believe are the most pressing challenges music recommender systems (MRS) are facing, from both academic and industry perspectives, and reviewed the state of the art toward solving these challenges and discussed their limitations. In order to solve the problems about the current existing data in online music service platforms which are heterogeneous, extensive, and disorganized, Lin et al. [11] proposed a heterogeneous knowledge-based attentive neural network model for short-term music recommendations, and the experimental results show that the proposed approach outperforms the current state-of-the-art short-term music recommendation systems on one real-world dataset. In addition, it can also recommend more relatively unpopular songs compared with classic models. Note recognition is the core and key aspect of music score recognition; Huang et al. [12] proposed an end-to-end detection model based on a deep convolutional neural network and feature fusion, and this model is able to directly process the entire image and then output the symbol categories and the pitch and duration of notes. Although the aforementioned research results can be innovative in the evaluation of symphony performance effect links, they still cannot effectively solve the intelligent analysis of performance effect evaluation and management [13–20].

The article "Audience Evaluation and Analysis of Symphony Performance Effects Based on the Genetic Neural Network Algorithm for the Multilayer Perceptron (GA-MLP-NN)" was retracted in 2023. Reasons: suspected computer-generated content; unreliable results or conclusions; concerns about the data; concerns about the results or conclusions.

In summary, it can be seen that most of the current orchestral music in performance effect analysis models does not involve an intelligent evaluation method based on performance effect and audience evaluation. In the evaluation of the delay effect of symphony in mainstream scientific research, most of researches are unified collection of data in the performance link, followed by postprocessing and analysis of the data, but rarely realize the “data collection” of the symphony performance link. Data analysis effect evaluation integrated real-time dynamic processing analysis. On the other hand, although the multilayer perceptual genetic neural network algorithm has been gradually applied in music evaluation, it has not been quickly and efficiently widely used in the stage of multianalysis and dynamic real-time processing of data. Therefore, it is important to study the orchestral performance effectiveness evaluation method based on multilayer perceptron genetic neural network algorithm.

## 3. Methodology

### 3.1. Ideas for the Application of Genetic Neural Network Algorithms for the Multilayer Perceptron Based on Mathematical Computation Theory

There are no more successful intelligent models applied in the world for studying optimization problems and simulation in the field of teaching quality assessment compared to genetic algorithms, particle swarm greedy algorithms, and local optimization neural network algorithms [21–26]. The multilayer perceptron genetic neural network algorithm (GA-MLP-NN) is based on the neural network algorithm and the genetic algorithm, combined with the correlation between the information and its fast optimization solution.

Based on this, in the orchestral performance effect analysis and evaluation model based on multilayer perceptron genetic neural network algorithm, the genetic neural network algorithm based on multilayer perceptron factors is firstly designed; that is, by combining neural network factors based on the level variability and audience evaluation effect in the process of orchestral performance, the quantitative evaluation of orchestral performance effect is realized. Then, the multilayer perceptron genetic neural network algorithm is used to precisely divide the information in a series of teaching processes expressed in the symphony performance analysis, so as to achieve a high degree of categorization of different qualities in the process of symphony performance analysis and melody research and to generate targets (symphony performance analysis pattern dividers) with a very high degree of synergistic correlation, which are pushed to the next stage of the process to be optimized to achieve a quantitative effect evaluation.

### 3.2. Construction of the Orchestral Performance Effect Evaluation Model Based on GA-MLP-NN Algorithm

In constructing the orchestral performance effect evaluation model and evaluation link based on the multilayer perceptron genetic neural network algorithm (GA-MLP-NN), the multilayer perceptron genetic neural network algorithm is used to categorize different types of symphonic music at different stages according to the similarity of vocal analysis patterns and the synergetic similarity of musical instruments, and then the melodic information in the analysis process of different symphonic performances is divided into secondary divisions, and, through the multilayer perceptron genetic neural network algorithm, the effect of symphonic performances of different degree types is selected for secondary division and update to ensure the stratification and update of effect analysis and management of different types of symphonic performances. Its data processing process is shown in Figure 1.

The article "Audience Evaluation and Analysis of Symphony Performance Effects Based on the Genetic Neural Network Algorithm for the Multilayer Perceptron (GA-MLP-NN)" was retracted in 2023. Reasons: suspected computer-generated content; unreliable results or conclusions; concerns about the data; concerns about the results or conclusions.

The steps are shown below.

In the first step, in the data analysis and processing link, the neural network data is classified according to the degree of association between the data and the difference of the modulus length after the data is vectorized, and a label is generated for each classified group for subsequent use. Supervised learning and then a neural network coding strategy are selected to transform the parameter set (feasible solution set) into a multilayer perceptron structure in a multilayer perceptron genetic neural network algorithm. In order to realize the process, this study combines a new multifactor coupling model-based orchestral performance process evaluation method, which uses the deformed coupling sequence to randomly displace common orchestral content and melody types, and then decouples it to achieve the optimal determination of different types of orchestral performance and performance process schemes and conducts simulation verification to evaluate this orchestral performance analysis quality evaluation scheme. It has a good objective evaluation capability. In this process, the simulation results of the relationship between the number of iterations of analysis and the coupled hierarchical perceptron are shown in Figure 2.

From Figure 2, it can be seen that, in the process of processing different data sets and averages under the multilayer perceptron genetic neural network algorithm, with the increase in the number of iterations of analysis, the change patterns of different coupling layer perceptrons are more obvious and similar in a certain range, which is because the multilayer perceptron genetic neural network algorithm follows the process of categorization of data before operation in the process of processing data. This is because the multilayer perceptron genetic neural network algorithm follows the rule of categorizing data before operation in processing data.

The expressions of the perceptual function *Q*(*x*), dimensional function *W*(*x*), and hierarchical function *E*(*x*) used in this process are given below, and they are often applied to some fields like image processing, image recognition, and image classification [27–31]:

(1) $$\begin{array}{c} Q\left(x\right)=\left(x^{2}+x+1\right)\frac{x\left(x+1\right)}{x+9},\\ W\left(x\right)=\left(\frac{3x^{2}+7x+1}{x+2}\right)\frac{\left(x-3\right)\left(x^{2}+1\right)}{x+3},\\ E\left(x\right)=\frac{\left(5x^{2}+7x+1/x+2\right)\left(\left(x-3\right)\left(x^{2}+1\right)/x+3\right)}{x+1+x^{-1}}, \end{array}$$

where *x* is the original input data. The results of the simulation analysis between different numbers of perceptrons and the number of neuron nodes in this stage are shown in Figure 3.

The article "Audience Evaluation and Analysis of Symphony Performance Effects Based on the Genetic Neural Network Algorithm for the Multilayer Perceptron (GA-MLP-NN)" was retracted in 2023. Reasons: suspected computer-generated content; unreliable results or conclusions; concerns about the data; concerns about the results or conclusions.

As can be seen in Figure 3, with the increase in the number of perceptrons under the multilayer perceptron genetic neural network algorithm, the change in the number of neuron nodes during the analysis of different database groups is different but the pattern is similar (all fall, then rise, and then fall), which is due to the formation of specific groups of vector matrices according to the difference in linguistic content and melodic variability of the orchestral performance audience evaluation method, and these matrices consist of different sets of vectors. These vector groups have different vector characteristic values according to the different similarity of the system's ability to analyze different symphony performances, thus realizing the conversion of the data of the same symphony performance analysis process into spatial vectors and digital information for storage and processing according to the expressiveness and existing level of language, and this process requires secondary analysis of the processed data; then the corresponding secondary perception function *Q*′(*x*), the true degree matching function *R*(*x*), and effect analysis function *T*(*x*) are expressed as

(2) $$\begin{array}{c} Q^{\prime }\left(x\right)=\left(\frac{x^{2}+x+1}{3x^{2}+2x+1}\right)\frac{x\left(x+1\right)}{x+9},\\ R\left(x\right)=\frac{3x^{2}+7x+1}{4x^{2}+9x+3},\\ T\left(x\right)=\frac{\left(6x^{2}+5x+3/x+3\right)}{x+1+x^{-1}}, \end{array}$$

where *x* is the original input data. The results of the simulation analysis of the relationship between the analysis strategy and the analysis quality factor for different dimensions in this stage are shown in Figure 4.

As can be seen in Figure 4, with the increase of dimensions in the analysis strategy under the multilayer perceptron genetic neural network algorithm, the difference in the change pattern of the analysis quality factor is more obvious in the process of analyzing different data information (4 sets of data types: 2 sets of training data and 2 sets of performance data), which is because the multilayer perceptron genetic neural network algorithm used in this study in processing the similar information is based on the different quality levels of different orchestral performance analysis patterns which are used as a basis to achieve a secondary division of different melodic types under the same orchestral performance analysis.

In the second step, a neural network node function is defined. We take a sequence of symphony types that conform to the algorithm rules *s*=(*c*_1_, *c*_2_,…, *c*_*n*_, *c*_*n*+1_). Thus, the neural network node function is

(3) $$\begin{array}{c} f\left(s\right)=\sum_{i=1}^{n}\frac{3s^{2}+5s+1}{s+1}. \end{array}$$

The basic implementation of this step is as follows: neuronal encoding of the individual *s*=(*c*_1_, *c*_2_,…, *c*_*n*_, *c*_*n*+1_) symphonic performance object. The results of performing layer 1, layer 2, layer 3, and layer 4 variants are

(4) $$\begin{array}{c} s_{1}={\sum_{1}^{m}\left(A,C,B,C,B,A\right)}^{m},\\ s_{2}={\overset{m+n}{\underset{1}{\sum }}\left(A,C,B,C,B,A\right)}^{m+n},\\ s_{3}={\sum_{1}^{m+2n}\left(B,A,B,C,C,A\right)}^{m+2n},\\ s_{4}={\sum_{1}^{m+3n}\left(B,B,C,C,A,A\right)}^{m+3n}, \end{array}$$

where (*A*, *B*, *C*) is the different variation rule. *m* is the *n*-dimensional information.

The article "Audience Evaluation and Analysis of Symphony Performance Effects Based on the Genetic Neural Network Algorithm for the Multilayer Perceptron (GA-MLP-NN)" was retracted in 2023. Reasons: suspected computer-generated content; unreliable results or conclusions; concerns about the data; concerns about the results or conclusions.

We then perform the regular recursive or neighborhood operation in the multilayer perceptron genetic neural network algorithm, such as swapping the last three, and then the variation results under 1, 2, 3, and 4 layer variation factors at this time are

(5) $$\begin{array}{c} s_{1}^{\prime }=\sqrt{{\sum_{1}^{m}\left(A,C,B,C,B,A\right)}^{m}},\\ s_{2}^{\prime }=\sqrt{{\sum_{1}^{m+n}\left(A,C,B,C,B,A\right)}^{m+n}},\\ s_{3}^{\prime }=\sqrt{{\sum_{1}^{m+2n}\left(B,A,B,C,C,A\right)}^{m+2n}},\\ s_{4}^{\prime }=\sqrt{{\sum_{1}^{m+3n}\left(B,B,C,C,A,A\right)}^{m+3n}}. \end{array}$$

The results of the simulation analysis of the relationship between different levels of variables and the effect evaluation index factors in this stage are shown in Figure 5.

As can be seen in Figure 5, under the multilayer perceptron genetic neural network algorithm, with the increase of layers in the variation factor, the effect evaluation index factors all show different degrees of fluctuating patterns in the process of analyzing different data information, which is caused by the inclusion type of the symphony set of the same spatial location stage as multiple pieces of evaluation data for the set operation.

### 3.3. Optimization Process of the Orchestral Performance Effect Evaluation Model Based on GA-MLP-NN Algorithm

In this orchestral performance effect evaluation model, in order to make different types of evaluation methods to maximize the evaluation level of different orchestral music types based on the existing melodic timbre and characteristic information status in the process of orchestral performance, the orchestral performance effect evaluation model is optimized by combining neural network algorithm and greedy optimization rules, and its optimization analysis process is shown in Figure 6.

The article "Audience Evaluation and Analysis of Symphony Performance Effects Based on the Genetic Neural Network Algorithm for the Multilayer Perceptron (GA-MLP-NN)" was retracted in 2023. Reasons: suspected computer-generated content; unreliable results or conclusions; concerns about the data; concerns about the results or conclusions.

The specific optimization process is divided into two steps.

First, the existing level information of common symphony types is first used to determine the appropriate recursion strategy according to the corresponding feature values and adaptations to achieve random generation of initialized neuron nodes. When the linguistic feature values of any two symphonies in the group are not the same, it means that the performance performative melodies of the two symphonies are extremely different, and automatic separation is achieved to calculate the number of symphonies in the group, perform the recursive postadaptation values, and compare them with the feature values and adaptations of the next target to be tested for analysis. When the multilayer perceptron genetic neural network algorithm is processed in deep mining for different symphonic performances, it generates different similarities in the types of symphonic melodies corresponding to the expression methods of the symphonic performances.

Second, in the optimization process of this multilayer perceptron genetic neural network algorithm-based orchestral performance effect evaluation model, the multilayer perceptron genetic neural network algorithm, in the actual evaluation process of a specific orchestral performance, transforms the timbral characteristics level information of the target orchestral performance type into computer-recognizable data information (such as vector groups and matrices) through specific processing, and then uses it in this process; the relationship between the different numbers of pointer patterns and the degree of difference of symphonic performance effect is shown in Figure 7.

As can be seen in Figure 7, with the increase of the number of evaluation dimensions in the pointer pattern under the multilayer perceptron genetic neural network algorithm, there are different degrees of changes among the orchestral performance effect evaluation indexes in the process of analyzing different types of data information, which is because the different pointer patterns will lead to large differences in the evaluation dimensions and will deepen the correlation between the data.

## 4. Result Analysis and Discussion

### 4.1. Experimental Design for the Validation of the Orchestral Performance Effect Evaluation Model

Assembling a comprehensive evaluation model based on symphonic performance analysis and symphonic performative melody analysis enables a more accurate assessment and analysis of the differences and characteristics of different types of symphonic music. Therefore, before conducting the experiment, a consistency assumption of noncore factors is required in order to reduce the interference of random factors.

The article "Audience Evaluation and Analysis of Symphony Performance Effects Based on the Genetic Neural Network Algorithm for the Multilayer Perceptron (GA-MLP-NN)" was retracted in 2023. Reasons: suspected computer-generated content; unreliable results or conclusions; concerns about the data; concerns about the results or conclusions.

In the experimental design link, this evaluation model can carry out feature monitoring when obtaining feature information of different orchestral performances, then realize feature information extraction from the monitored data, carry out further study through the analysis process of melodies and evaluation carriers in the process of multiple orchestral performances, and, finally, through data analysis of dynamic detection and experimental process, compare with the feature values of the standardized analysis model to realize in evaluation in terms of core indicators. The format of the input data in this experimental process and the previous simulation analysis process is the data matrix filled by the quantitatively evaluated data vector group, which uses the function of how to extract the input data. The dimensions of the data matrix are dynamically adjusted (so that the calculation time can be adaptively optimized). The input layer, hidden layer, and output layer have an upper limit of 100 nodes. In addition, the data intervals in terms of crossover rate and data mutation rate are both 0.2–1.0.

In the evaluation session, the stored information about the characteristics of the symphony in terms of language and melody will be stored for further comprehensive evaluation of the quality of different vocal music analysis modes at a later stage, so as to achieve an intelligent analysis of the quality of symphony performance analysis and thus an objective evaluation under the innovative mode of symphony performance analysis based on the multilayer perceptron genetic neural network algorithm.

According to the multiple influential indicators, it is possible to achieve the optimization and high-quality development of each vocal music analysis model scheme, to quickly enhance the data recording for each symphony type, and thus to achieve intelligent recording for different students. This orchestral performance evaluation model analyzes four indicators (orchestral performance type, melodic characteristics, audience evaluation, and performance effect) for the first group of objects and the second group of objects, and the experimental analysis results of the deep recursive processing of neural networks at different levels are shown in Figure 8.

As can be seen in Figure 8, under the multilayer perceptron genetic neural network algorithm, the evaluation efficiency of the experimental data is also significantly improved with the increase of the number of neural network layers at three different threshold factors (0.1/0.5/1.0), which is because the increase of the neural network layers leads to an increase of the maximum dimensionality of the data analysis and at the same time makes the rate of single processing data increase, so the overall evaluation efficiency is also faster. On the other hand, as the number of layers of the neural network changes, its internal data relevance also has varying degrees of coupling changes, and the changes in the three thresholds can well produce more relevance to different data. Therefore, as the number of neural network layers increases, its evaluation efficiency is also significantly improved.

The article "Audience Evaluation and Analysis of Symphony Performance Effects Based on the Genetic Neural Network Algorithm for the Multilayer Perceptron (GA-MLP-NN)" was retracted in 2023. Reasons: suspected computer-generated content; unreliable results or conclusions; concerns about the data; concerns about the results or conclusions.

### 4.2. Experimental Results and Analysis

The comparison results of the objective indexes for the evaluation of orchestral performance effects combining multilayer perceptron genetic neural network algorithm and intelligent fuzzy evaluation are shown in Table 1.

The analysis of the error degree of the results during the experiment under the multilayer perceptron genetic neural network algorithm is shown in Figure 9.

From Figure 9, it can be seen that the error degrees of orchestral performance effects analyzed by different methods under the multilayer perceptron genetic neural network algorithm are different, and they all show different trends. Compared with the GA-NN method and the MLP-NN method, the GA-MLP-NN method obtained the smallest error and the highest accuracy, and the error can be controlled within the effective range in less than 8 times of analysis, so the GA-MLP-NN method has better evaluation stability.

Therefore, combining the results of Figure 9, according to the experimental results, it is possible to analyze the improvement of performance analysis and audience evaluation of one random symphony (the extraction process is between 20% and 80% from the center of the spatial location, and random numbers are used for irregular extraction) as a control experiment, where one symphony starts with a moderately low level of performance analysis and audience evaluation (ranking in the combined level). Through the application of multilayer perceptron genetic neural network algorithm and fuzzy evaluation of orchestral performance effect analysis model, it was found that the experimental group and the control group had a great improvement in performance effect analysis and audience evaluation. One improved from ranking outside 75.3% in the group in terms of overall analysis effect to within 30.1%. The other orchestral performance effect improved from within 15.4% to within 12.8% of the overall analysis effect ranking in the audience group. This shows that the present orchestral performance effect evaluation management and analysis model based on multilayer perceptron genetic neural network algorithm is capable of quantitative evaluation and multidimensional analysis of orchestral performance effect, which is of practical significance to the innovation and application of orchestral performance effect evaluation management nowadays.

The article "Audience Evaluation and Analysis of Symphony Performance Effects Based on the Genetic Neural Network Algorithm for the Multilayer Perceptron (GA-MLP-NN)" was retracted in 2023. Reasons: suspected computer-generated content; unreliable results or conclusions; concerns about the data; concerns about the results or conclusions.

## 5. Conclusion

In order to better realize the quantitative evaluation enhancement of symphony performance effect, the innovation of the current symphony performance effect evaluation and analysis model in China is imperative. Based on this, this paper uses genetic neural network algorithm based on multilayer perceptron and fuzzy evaluation model and firstly selects three characteristic parameters related to symphony performance-related analysis and proposes an evaluation system based on the characteristic parameters of symphony performance effect. This orchestral performance effect evaluation model is evaluated from multiple perspectives by studying the type of orchestral performance, vocal playing ability, vocal coordination ability, audience evaluation effect, and timbre feature extraction analysis in the analysis process. The final experimental results show that the use of multilayer perceptron genetic neural network algorithm to characterize the effectiveness of the innovation model can achieve comprehensive evaluation. However, this study did not evaluate the effectiveness of specific types of orchestral performances in a targeted manner, so in-depth research can be conducted on the scope of application and customized analysis.

## Figures and Tables

**Figure 1:** Data analysis and processing process of GA-MLP-NN algorithm.

**Figure 2:** The relationship between the number of iterations of analysis and the coupling level perceptron under the GA-MLP-NN algorithm.

**Figure 3:** Simulation of the relationship between different numbers of perceptrons and the number of neuron nodes.

**Figure 4:** Simulation of the relationship between the analysis strategy of different dimensions and the analysis quality factor under the GA-MLP-NN algorithm.

**Figure 5:** The simulation analysis results of the relationship between the variation factors of different levels and the effect evaluation index factors.

**Figure 6:** Optimization model of symphony performance evaluation based on GA-MLP-NN algorithm.

**Figure 7:** Simulation analysis results of the relationship between different numbers of pointer modes and the degree of difference in symphony performance.

**Figure 8:** Experimental analysis results of deep recursive processing of neural networks at different levels.

**Figure 9:** Analysis of the error degree of the results during the experiment.

**Table 1:** Comparison of different evaluation indicators under different methods.

Evaluation index	Multilayer perceptron genetic neural network algorithm	Other mainstream quantitative evaluation algorithms
Evaluation accuracy (%)	>95.3	>91.1
Evaluation error rate (%)	<3.4	<5.8

The article "Audience Evaluation and Analysis of Symphony Performance Effects Based on the Genetic Neural Network Algorithm for the Multilayer Perceptron (GA-MLP-NN)" was retracted in 2023. Reasons: suspected computer-generated content; unreliable results or conclusions; concerns about the data; concerns about the results or conclusions.

## Data Availability

The data used to support the findings of this study are available upon request to the author.
